The article "An Antioxidant Extract of Tropical Lichen,Parmotrema reticulatum, Induces Cell Cycle Arrest and Apoptosis in Breast Carcinoma Cell Line MCF-7" was published in 2013. Journal: PLoS One.

# An Antioxidant Extract of Tropical Lichen,*Parmotrema reticulatum*, Induces Cell Cycle Arrest and Apoptosis in Breast Carcinoma Cell Line MCF-7

**DOI:** 10.1371/journal.pone.0082293

**Published:** 2013-12-16

**Authors:** Nikhil Baban Ghate, Dipankar Chaudhuri, Rhitajit Sarkar, Albert L. Sajem, Sourav Panja, Jayashree Rout, Nripendranath Mandal

**Affiliations:** 1 Division of Molecular Medicine, Bose Institute, Kolkata, India; 2 Department of Ecology and Environmental Science, Assam University, Silchar, Assam, India; Indian Institute of Toxicology Reserach, India

## Abstract

This report highlights the phytochemical analysis, antioxidant potential and anticancer activity against breast carcinoma of 70% methanolic extract of lichen, *Parmotrema reticulatum* (PRME). Phytochemical analysis of PRME confirms the presence of various phytoconstituents like alkaloids, carbohydrates, flavonoids, glycosides, phenols, saponins, tannins, anthraquinones, and ascorbic acid; among which alkaloids, phenols and flavonoids are found in abundant amount. High performance liquid chromatography (HPLC) analysis of PRME revealed the presence of catechin, purpurin, tannic acid and reserpine. Antioxidant activity was evaluated by nine separate methods. PRME showed excellent hydroxyl and hypochlorous radical scavenging as well as moderate DPPH, superoxide, singlet oxygen, nitric oxide and peroxynitrite scavenging activity. Cytotoxicity of PRME was tested against breast carcinoma (MCF-7), lung carcinoma (A549) and normal lung fibroblast (WI-38) using WST-1 method. PRME was found cytotoxic against MCF-7 cells with an IC_50_ value 130.03±3.11 µg/ml while negligible cytotoxicity was observed on A549 and WI-38 cells. Further flow cytometric study showed that PRME halted the MCF-7 cells in S and G2/M phases and induces apoptosis in dose as well as time dependent manner. Cell cycle arrest was associated with downregulation of cyclin B1, Cdk-2 and Cdc25C as well as slight decrease in the expression of Cdk-1 and cyclin A1 with subsequent upregulation of p53 and p21. Moreover PRME induced Bax and inhibited Bcl-2 expression, which results in increasing Bax/Bcl-2 ratio and activation of caspase cascade. This ultimately leads to PARP degradation and induces apoptosis in MCF-7 cells. It can be hypothesised from the current study that the antioxidant and anticancer potential of the PRME may reside in the phytoconstitutents present in it and therefore, PRME may be used as a possible source of natural antioxidant that may be developed to an anticancer agent.

## Introduction

The free radicals are generated in various biological systems and also in the human body in the form of reactive oxygen species (ROS) and reactive nitrogen species (RNS). These free radicals cause cellular injury which is associated with aging and over 200 clinical disorders including cancer, heart disease, liver damage, neurodegenerative diseases and other degenerative diseases related to inflammation [1]. Antioxidants, possible protective agents, can be considered to ease from oxidative damage caused by free radicals in the human body and retarding the progress of many chronic diseases including ageing and cancer [2]–[4]. These natural antioxidants could modify the behaviour of cancer cells by altering their redox environment [5], [6] as well as reduce their genetic instability and thus may be considered useful in cancer treatment [7]. The mechanism by which antioxidants improve the efficacy of chemotherapy is also demonstrated previously [8]. Worldwide, Breast cancer is the most common cause of cancer-related death in women with 4,58,000 deaths annually. While lung cancer, causes death both in men and women, is responsible for 1.3 million deaths annually, as on 2004 [9]. Several strategies are involved in combating cancer, chemotherapy is getting more importance and occurring effective against most of the cancer types but the drug resistance limits successful outcomes in most cases. Moreover, the drugs’ inability to distinguish between normal and cancerous cells make hinders their unanimous choice. Thus major attention is being given to search for better and safer antioxidants of natural origin, which may raise the efficiency of cancer treatment.

Recently, much attention has been paid to several lichen species as resources of natural antioxidants. Lichens are the symbiotic products of the mycobiont (fungal partner) and photobiont (algal partner). Lichens produce a varied range of secondary metabolites and also some of them are unique to lichen symbiosis including depsides, depsidones, dibenzofurans and pulvinic acid. These compounds have attracted much attention in investigations because of their antiviral, antibiotic, antioxidant, antitumor, allergenic and plant growth inhibitory activities [10]–[12]. Previously many lichens have been reported for their antimicrobial [13]–[15], antioxidant [16]–[18] and anticancer [18]–[20] properties. The genus *Parmotrema* is typically characterized by large foliose thalli with broad lobes, commonly with a broad marginal zone on the lower surface, pored epicortex, thick-walled hyaline ellipsoid ascospores, sublageniform or filiform conidia and with or without marginal cilia. The greatest distribution of the genus is in tropical regions, where more than 220 species found out of 350 known species [21]. Several species of *Parmotrema* have also reported for their diverse and potent pharmacological activities like antimicrobial [22]–[26] and antioxidant [27] properties. *Parmotrema reticulatum* occur in abundance in Dima Hasao Hills district of Assam, North-East, India. This species has been preliminary screened for its antioxidant [28] and antibacterial [29] activities. Even though these manifold activities of the lichen have now been recognized, their therapeutic potential remains unexploited. Hence this work was set out in order to establish the antioxidant activity as well as anticancer potential against lung and breast carcinoma of 70% methanolic extract of *P. reticulatum* (PRME) using A549 and MCF-7 as a model cell lines.

## Materials and Methods

### Chemicals

2,2′-azinobis-(3-ethylbenzothiazoline-6-sulfonic acid) (ABTS), Cell Proliferation Reagent WST-1, Annexin-V-FLUOS staining kit and Polyvinyl difluoride membrane was procured from Roche diagnostics, Mannheim, Germany. 6-hydroxy-2,5,7,8-tetramethylchroman-2-carboxylic acid (Trolox) was obtained from Fluka, Buchs, Switzerland. Potassium persulfate (K_2_S_2_O_8_), 2-deoxy-2-ribose, ethylene diammine tetraacetic acid (EDTA), ascorbic acid, trichloroacetic acid (TCA), mannitol, nitro blue tetrazolium (NBT), reduced nicotinamide adenine dinucleotide (NADH), phenazine metho-sulfate (PMS), sodium nitroprusside (SNP), 1,10-phenanthroline, sulphanilamide, naphthyl ethylenediamine dihydrochloride (NED), L-histidine, lipoic acid, sodium pyruvate, quercetin and ferrozine were obtained from Sisco Research Laboratories Pvt. Ltd, Mumbai, India. HPLC grade acetonitrile, ammonium acetate, hydrogen peroxide, potassium hexacyanoferate, Folin-ciocalteu reagent, sodium carbonate, mercuric chloride, potassium iodide, anthrone, vanillin, thiourea, 2,4-dinitro-phenylhydrazine, sodium hypochlorite, aluminium chloride, xylenol orange, butylated hydroxytoluene (BHT), N,N- dimethyl-4-nitrosoaniline and BCIP/NBT substrate were taken from Merck, Mumbai, India. 1,1-diphenyl-2-picrylhydrazyl (DPPH), gallic acid, (+) catechin, curcumin, RNAase A, 4′,6′-diamidino-2 phenylindole and Triton X-100 were obtained from MP Biomedicals, France. Catalase, reserpine, sodium bicarbonate Ham’s F-12, Dulbecco’s Modified Eagle’s Medium (DMEM), antibiotics and Amphotercin-B were obtained from HiMedia Laboratories Pvt. Ltd, Mumbai, India. Evans blue was purchased from BDH, England. D-glucose was procured from Qualigens Fine Chemicals, Mumbai. Diethylene-triamine-pentaacetic acid (DTPA) was obtained from Spectrochem Pvt. Ltd, Mumbai, India. Thiobarbituric acid (TBA) was obtained from Loba Chemie, Mumbai, India. Fetal bovine serum was purchased from HyClone Laboratories, Inc., Utah, USA. Non-Fat dry milk was purchased from Mother Dairy, G. C. M. M. F. Ltd. AMUL, India. Anti-Bcl-2 (NT), anti-Caspase-9 and anti-p53 antibodies were purchased from AnaSpec, Inc., USA. Anti-PARP, anti-caspase-3, anti-caspase-8, anti-Bax, anti-BID and anti-beta-actin antibodies were purchased from OriGene technologies, Inc, Rockville, USA. Anti-Cyclin A1, anti-Cyclin B1, anti-Cdc25C, anti-CDK2, anti-CDK1 were purchased from Bioss, Inc., Woburn, USA. Anti-p21 (WAF1, Cip1) was purchased from eBioscience San Diego, USA. Alkaline phosphatase conjugated anti-Rabbit secondary antibody was purchased from RockLand immunochemicals Inc., Gilbertsville, USA.

### Ethics

The lichen sample of *Parmotrema reticulatum* (Taylor) M. Choisy was collected from some home gardens or public areas adjoining some villages in Dima Hasao Hills district, Assam, India. These areas are not within a National Park/Reserve Forest/Govt. protected area, only verbal permissions from village headmen were obtained before collection. The conservation status of this lichen was classified using the International Union for Conservation of Nature (IUCN) World Conservation Union guidelines (1994). Status: EN (D); Endangered, as per IUCN red list criteria. The material collected for this study was only sampled at a very limited scale and therefore had negligible effects on broader ecosystem functioning.

### Sample Extraction and Preparation

The lichen was identified based on morphologoical, anatomical and chemical analysis following keys [30], [31]. The morphology and anatomy of the thallus was studied using an optical microscope and chemical test was performed by spot tests and thin layer chromatography (TLC). Samples were sorted, cleaned of substratum and dried for extraction. The air-dried sample (100 g) was then powdered and stirred using a magnetic stirrer with 70% methanol in water (1000 ml) for 15 hours; the mixture was then centrifuged at 2850×*g* and the supernatant was decanted. The process was repeated by adding the same solvent with the precipitated pellet. The supernatants from two phases were mixed, concentrated in a rotary evaporator at 40°C and lyophilized. The obtained dried extract was stored at −20°C until use. For antioxidant studies PRME was dissolved at a concentration of 1 mg/ml in water and for anticancer studies working stock solution (2 mg/ml) was prepared in 0.25% DMSO in water and sterilised using 0.22 µm syringe filter.

### Standardisation of the Lichen Extract

The analysis of resident phytochemicals like alkaloids, carbohydrates, flavonoids, glycosides, phenols, saponins, tannins, terpenoids, anthraquinones and triterpenoids in the extract was carried out using standard qualitative and quantitative methods as described previously [32], [33].

#### HPLC standardisation of the lichen extract

For HPLC analysis, stock solutions (10 µg/ml) were prepared in mobile phase for the sample (PRME) and gallic acid, catechin, reserpine, quercetin and tannic acid as standards. Samples were then filtered through 0.45 µm polytetrafluoroethylene (PTFE) filter (Millipore) to remove any particulate matter. Analysis was performed using a HPLC-Prominence System RF10AXL (Shimadzu Corp.) equipped with degasser (DGU-20A5), quaternary pump (LC-20AT), auto-sampler (SIL-20A) and detectors of Reflective Index (RID-10A), Fluorescence (RF-10AXL) and Diode Array (SPD-M20A). 20 µl of sample and standards were injected and analyzed in triplicates. Gradient elution consecutive mobile phases of acetonitrile and 0.5 mM ammonium acetate in water, at a flow rate of 1 ml/min for 65 min through the column (Z1C-HILIC) that was maintained at 25°C. The detection was carried out at 254 nm.

### *In Vitro* Antioxidant and Free Radical Scavenging Activity

#### Total antioxidant activity

Total antioxidant capacities of the extract were evaluated by ABTS**•** ^+^ radical cation decolourisation assay in comparison to trolox standard [34] and DPPH radical scavenging assay [35].

#### Reactive oxygen species (ROS) scavenging activity

*In vitro* ROS scavenging property of the extract was determined by different stable ROS radical scavenging assays such as hydroxyl, superoxide, hypochlorous radical and singlet oxygen assays by standard procedures [34].

#### Reactive nitrogen species (RNS) scavenging activity

RNS Scavenging activity of the extract was determined by nitric oxide and peroxynitrite radical scavenging assays [34].

### *In Vitro* Anticancer Study

#### Cell lines and culture

Human lung adenocarcinoma (A549), human breast adenocarcinoma (MCF-7) and human lung fibroblast (WI-38) cell line were purchased from the National Centre for Cell Science (NCCS), India and maintained in the laboratory. A549 cells were grown in Ham’s F-12 medium whereas MCF-7 and WI-38 cells were grown in DMEM. Both the media were supplemented with 10% (v/v) fetal bovine serum (FBS), 100 U/ml Penicillin G, 50 µg/ml Gentamycin sulphate, 100 µg/ml Streptomycin and 2.5 µg/ml Amphotericin B. All the cell lines were maintained at 37°C in a humidified atmosphere containing 5% CO_2_ in CO_2_ incubator.

#### WST-1 cytotoxicity assay

Cell proliferation and cell viability were quantified using the WST-1 Cell Proliferation Reagent, Roche diagnostics, according to the previously described method [36]. In brief, A549, MCF-7 and WI-38 cells (1×10^4^ cells/well) were treated with PRME, tannic acid, catechin, purpurin and reserpine ranging from 0–300 µg/ml for 48 hours in 96-well culture plate. After treatment, 10 µl of WST-1 cell proliferation reagent was added to each well followed by 2 hours of incubation at 37°C. Cell proliferation and viability were quantified by measuring absorbance at 460 nm using a microplate ELISA reader MULTISKAN EX (Thermo Electron Corporation, USA).

#### Cell cycle analysis

Cell cycle analysis was performed by flow cytometry using the method previously described [36]. MCF-7 cells (1×10^6^) were treated with PRME (0–300 µg/ml) for 48 hours and the same number of the cells were treated with PRME (300 µg/ml) for different time intervals (0–48 hours). After treatment, nuclear DNA of cells was then stained with propidium iodide and cell phase distribution was determined on FACS Verse (Becton Dickinson) equipped with 488 nm (Blue), 405 nm (Violet) and 640 nm (Red) solid state laser light using FACSuite software Version 1.0.3.2942. A total 10000 events were acquired and data analysis was done using the same software. A histogram of DNA content (x-axis, red fluorescence) vs count (y- axis) was plotted.

#### Annexin V staining

This assay was performed using Annexin-V-FLUOS Staining kit, Roche diagnostics. MCF-7 cells (1×10^6^) were treated with PRME (0–300 µg/ml) for 48 hours and the same number of the cells were treated with PRME (300 µg/ml) for different time intervals (0–48 hours). After treatment cells were labelled with PI and FITC according to the protocol of the kit manufacturer. The distribution of apoptotic cells was identified by flow cytometer on FACS Verse (Becton Dickinson) equipped with 488 nm (Blue), 405 nm (Violet) and 640 nm (Red) solid state laser light using FACSuite software Version 1.0.3.2942. A total 10000 events were counted. Cells that were Annexin V (−) and PI (−) were considered as viable cells. Cells that were Annexin V (+) and PI (−) were considered as early stage apoptotic cells. Cells that were Annexin V (+) and PI (+) were considered as late apoptotic or necrotic cells.

#### Western blot analysis

1×10^6^ MCF-7 cells were treated with PRME (300 µg/ml) for various time intervals (6–48 hours). After treatment, cells were lysed with triple detergent cell lysis buffer (50 mM Tris-Cl, 150 mM NaCl, 0.02% Sodium azide, 0.1% Sodium dodecyl sulphate, 1% triton X-100, 0.5% sodium deoxycholate, 1 µg/ml aprotinin, 100 µg/ml phenyl methyl-sulfonyl fluoride, pH 8) and the lysates were then centrifuged at 13800×*g* for 20 minutes at 4°C. Protein concentration was measured by Folin-Lowry method. Proteins (40 µg) in the cell lysates were resolved on 12% SDS-PAGE and transferred to the PVDF membrane using transfer buffer (39 mM Glycine, 48 mM Tris base, 20% Methanol, 0.037% Sodium dodecyl sulphate, pH 8.3). The membranes were then blocked with 5% non-fat dry milk in TBS followed by incubation with corresponding antibodies separately overnight at 4°C. After washing with TBS-T (0.01% of Tween-20 in TBS) membranes were incubated with alkaline phosphatase conjugated anti-Rabbit IgG antibody at room temperature in the dark for 4 hours, followed by washing. The blots were then developed with BCIP/NBT substrate and the images were taken by the imaging system EC3 Chemi HR (UVP, USA). The blots were then analysed for band densities using ImageJ 1.45s software.

#### Statistical analysis

All spectrophotometric data were data was reported as the mean ± SD of 6 measurements and cell cycle analysis data was reported as the mean ± SD of 3 measurements. The statistical analysis was performed by KyPlot version 2.0 beta 15 (32 bit). The IC_50_ values were calculated by the formula, Y = 100*A1/(X+A1) where A1 =  IC_50_, Y = response (Y = 100% when X = 0), X = inhibitory concentration. The IC_50_ values were compared by paired *t*-test. P<0.05 was considered significant.

## Results and Discussion

### PRME Acts as a Effective Antioxidant and Free Radical Scavenger

Antioxidants are the compounds or systems that inhibit formation of free radicals or interrupt propagation of the same by one (or more) of several mechanisms [37]. Total antioxidant activity of the extract (PRME) was calculated, and as a function of the trolox (standard) equivalent antioxidant capacity (TEAC) was found to be 0.417±0.012 (Table 1). The hydroxyl radical, one of the reactive free radicals formed in biological systems, causes enormous damage on biomolecules of the living cells [38]. Another harmful ROS is hypochlorous acid and it is produced at the sites of inflammation by the oxidation of Cl¯ ions by the neutrophil enzyme myeloperoxidase [39]. PRME showed excellent dose dependent hydroxyl radical (Figure 1A) as well as hypochlorous radical (Figure 1B) scavenging activity than the respective standard compounds. DPPH is a stable free radical and accepted widely as a system for estimating antioxidative capacity. Singlet oxygen, a high energy form of oxygen, was generated in the skin upon UV-radiation and induces hyperoxidation, oxygen cytotoxicity and decreases the antioxidant activity [40]. Likewise, superoxide anion is also considered as one of the harmful reactive oxygen species. PRME moderately scavenged superoxide (Figure 1C), singlet oxygen radicals (Figure 1D). and DPPH (Figure 2). IC_50_ values of PRME on different radical scavenging were shown in Table 1 with their respective standard compounds. The production of nitric oxide radical at a sustained level results in direct tissue toxicity and contribute to the vascular collapse associated with septic shock, whereas chronic expression of nitric oxide radical is associated with various carcinomas and inflammatory conditions including juvenile diabetes, multiple sclerosis, arthritis and ulcerative colitis [41]. Moreover, the toxic effect of NO increases greatly upon reaction with superoxide radical and resulting in formation of highly reactive peroxynitrite anion (ONOŌ). In the present study, it was found that PRME showed moderate scavenging activity against both nitric oxide (Figure 3A) and peroxynitrite radicals (Figure 3B). IC_50_ values of PRME on both the radical scavenging were shown in Table 1 with their respective standard compounds.

**Figure 1:** Reactive Oxygen species scavenging activity of PRME and the reference compounds. (A) Hydroxyl radical inhibition, (B) hypochlorous radical scavenging, (C) superoxide radical inhibition, (D) singlet oxygen radical scavenging. The results are mean ± S.D. of six parallel measurements. **p<0.01 and ***p<0.001 vs. 0 µg/ml.

**Figure 2:** DPPH radical scavenging activity of PRME and the reference compound. The results are mean ± S.D. of six parallel measurements. **p<0.01 and ***p<0.001 vs. 0 µg/ml.

**Figure 3:** Reactive Nitrogen species scavenging activity of PRME and the reference compounds. (A) Nitric oxide inhibition, (B) peroxynitrite radical scavenging. The results are mean ± S.D. of six parallel measurements. ***p<0.001 vs. 0 µg/ml.

**Table 1:** Trolox equivalent antioxidant capacity and IC_50_ values of the lichen extract (PRME) and standard compounds for ROS and RNS scavenging.

Name of Assay	PRME	Standard	Values of Standard compounds
TEAC Values	0.417±0.012	**–**	**–**
#IC_50_ values of the extracts for free radical scavenging capacity for			
DPPH	311.75±25.02***	Ascorbic acid	5.29±0.28
Hydroxyl radical (OH^•^) scavenging	73.83±1.09***	Mannitol	571.45±20.12
Superoxide anion (O_2_^•−^) scavenging	241.68±1.19***	Quercetin	42.06±1.35
Nitric oxide radical (NO) scavenging	416.39±12.57***	Curcumin	90.82±4.75
Peroxynitrite (ONOO^−^) scavenging	3.852±0.27***	Gallic acid	0.876±0.57
Singlet oxygen (^1^O_2_) scavenging	0.545±0.01***	Lipoic acid	0.046±0.01
Hypochlorous acid (HOCl) scavenging	55.09±0.97***	Ascorbic acid	235.96±5.75

_50_ values of all activities are determined in µg/ml. Data expressed as mean ± S.D (n = 6). EDTA represents Ethylenediamine tetraacetic acid.^#^ IC

p<0.001.

### PRME Inhibits Growth of Breast Cancer MCF-7 Cells but Not Lung Cancer A549 and Non-malignant WI-38 Cells

There are numerous reports on the positive correlation between antioxidant activities and cytotoxicity of compounds from plant, viz. resveratrol, quercetin, selenium and vitamin E, towards cancer cell [42], [43]. The cytotoxicity of PRME on lung (A549) and breast (MCF-7) carcinoma as well as one non-malignant cell line (WI-38) was performed using WST-1 assay; the results are shown in Figure 4. PRME was found cytotoxic to MCF-7 cell and inhibited its growth in a dose dependent manner with an IC_50_ value of 130.03±3.11 µg/ml. However, the presence of PRME did not inhibit the cell proliferation of A549 and WI-38 cells significantly and IC_50_ values were found 773.62±88.39 µg/ml and 826.53±90.34 µg/ml, respectively. This result indicates that PRME has *in vitro* anticancer activity against breast carcinoma (MCF-7) but not against lung carcinoma (A549) and also not toxic to the normal lung fibroblast cells (WI-38).

**Figure 4:** Effect of PRME on cell proliferation and viability of A549, MCF-7 and WI-38 cells. Cells were treated with increasing concentrations of PRME for 48 hours; cell proliferation and viability was determined with WST-1 cell proliferation reagent. Results were expressed as cell viability (% of control). All data is expressed as mean ± SD (n = 6). *p<0.05, **p<0.01 and ***p<0.001 vs. 0 µg/ml.

### PRME Induces S and G2/M Phase Arrest and Apoptosis in MCF-7 Cells

Many anticancer agents arrest the cell cycle at G0/G1, S and G2/M phase and then induce apoptosis [44], [45] or directly induce apoptosis to kill cancer cell [46]. The effect of PRME on cell cycle distribution of MCF-7 cells was studied to verify the mechanism by which anticancer effect was achieved. PRME arrested the MCF-7 cells in both G2/M phase and to a lesser extent in S phase in a dose dependent manner with an effective arrest at a dose of 300 µg/ml. This accumulation of cells in S and G2/M phase also coincides with the occurrence of Sub-G1 population which refers to apoptotic cells (Figure 5). Furthermore, to confirm the dose dependent induction of apoptosis in MCF-7 cells, Annexin-V staining was performed (Figure 6). It was observed that the treatment of PRME with increasing doses leads to the increase in apoptotic cells. At concentration of 200 µg/ml both early (72.94%) and late apoptotic cells (18.00%) were found however, when MCF-7 cells were treated with higher dose of PRME (300 µg/ml) it was observed that the late apoptotic population (22.82%) was increased which indicates that the higher dose of PRME is effective in killing MCF-7 cells by inducing apoptosis. Likewise, incubation of MCF-7 cells with an extract concentration of 300 µg/ml for various time intervals also found to increase the S and G2/M phase arrest in a time dependent manner (Figure 7). Alongside, time dependent increase in early apoptotic cells was observed when MCF-7 cells were treated with PRME (300 µg/ml). At 6 hours 9.11%, at 12 hours 19.81%, at 24 hours 25.18% and at 36 hours 68.19% of cells were found in early apoptotic stage. The incubation of cells with PRME for additional time (48 hours) results in increase in the late apoptotic cells (19.03%) (Figure 8). Thus, results from flow cytometric studies suggest that PRME induced S and G2/M phase arrest as well as apoptosis in dose and time dependent manner.

**Figure 5:** Flow cytometric cell cycle distribution of PRME treated MCF-7 cells with increasing doses. Sub-G1, G1, S, and G2/M phases of MCF-7 cells treated for 48 hours with different concentrations: (A) Control, (B) 50 µg/ml, (C) 80 µg/ml, (D) 100 µg/ml, (E) 200 µg/ml, (F) 300 µg/ml of PRME. (G) Graphical representation of % cell population in different phases.

**Figure 6:** Flow cytometric plots of Annexin-V-FLUOS and PI staining of PRME treated MCF-7 cells with increasing doses. MCF-7 cells were treated for 48 hours with different concentrations: (A) Control, (B) 50 µg/ml, (C) 80 µg/ml, (D) 100 µg/ml, (E) 200 µg/ml, (F) 300 µg/ml of PRME. Numbers in boxes represent % of total cells in respective boxes.

**Figure 7:** Flow cytometric cell cycle distribution of PRME treated MCF-7 cells with increasing time. Sub-G1, G1, S, and G2/M phases of PRME (300 µg/ml) treated MCF-7 cells at (A) 0 hour, (B) 6 hours, (C) 12 hours, (D) 24 hours, (E) 36 hours, (F) 48 hours. (G) Graphical representation of % cell population in different phases.

**Figure 8:** Flow cytometric plots of Annexin-V-FLUOS and PI staining of PRME treated MCF-7 cells with increasing time. MCF-7 cells were treated with PRME (300 µg/ml) for different time intervals: (A) 0 hour, (B) 6 hours, (C) 12 hours, (D) 24 hours, (E) 36 hours, (F) 48 hours. Numbers in boxes represent % of total cells in respective boxes.

### PRME Regulates the Expression of Various Cell Cycle Related Proteins and Activates Tumor Suppressor p53 in MCF-7 Cells

We next examined the effect of PRME for expression of various cell cycle related proteins. Results showed that PRME inhibited the expression of almost all the cell cycle related proteins which we have studied. The expression of cyclin B1 (Figure 9A), Cdk-2 (Figure 9B) and Cdc25C (Figure 9C) was decreased dramatically with time. However, the expression of Cdk-1 (Figure 9D), cyclin A1 (Figure 9E) was not inhibited that much, which allows some cells to transit from S phase to G2 phase. It is known that cyclin B1/Cdk-1 complex and cyclin A1/Cdk-2 complex are important for G2-M phase transition and S-G2 phase transition respectively [47]. p53 is a tumor suppressor protein and has been shown to play a key role in the regulation of cell cycle and apoptosis. Several stresses such as DNA damage may lead to the activation of p53 and results in the arrest of cell cycle at G0/G1, S or G2/M phase by activating its target genes especially p21 or by inhibiting cyclins and Cdks directly [48], [49]. The involvement of p53 and its downstream Cdk inhibitor p21 in PRME-treated MCF-7 cells was then investigated. The study showed that the protein levels of p53 (Figure 9F) and p21 (Figure 9G) increased significantly with increasing exposure time to PRME. These results indicate that a p53-dependent cascade signalling pathway was involved in the PRME modulation of the cell-cycle machinery of MCF-7 cells.

**Figure 9:** Western blot analysis of cell cycle related proteins of MCF-7 cells treated with 300 µg/ml PRME. Graphs adjoining the blots represent the expression levels of corresponding proteins for indicated time intervals: (A) Cyclin B1, (B) Cdk-2, (C) Cdc25c, (D) Cdk-1, (E) Cyclin A1, (F) p53, (G) p21.

### PRME Regulates the Expression of Bcl-2 Family Proteins and Activates Caspase Cascade in MCF-7 Cells

Two major mechanisms exist that induce apoptosis by initiating the caspase cascade: the extrinsic pathway involving caspase-8; and the intrinsic pathway involving caspase-9 as the initiator caspase. Expressed as inactive enzymes, caspases are members of a family of cysteine proteases, play a central role in apoptosis [50]. Once activated, caspase-8 activates the downstream executioner caspase-3 by proteolytic cleavage of its zymogen form. The other initiator caspase, caspase-9, respond to the release of cytochrome C from the mitochondria. Once released from mitochondria, cytochrome C acts as a co-factor and interacts with Apaf-1 and procaspase-9, which in turn activates caspase-9. This formed apoptosome is then involved in the activation of caspase-3. Activated caspase-3 is responsible for the proteolytic degradation of PARP, which occurs at the onset of apoptosis [51]. PRME treated and untreated MCF-7 cells were further analysed for the expression of apoptosis related proteins. It is found from the results that the expression levels of pro-caspases-3, and 9 is decreased with increase in the levels of cleaved caspase-9, and 3; as well as degradation of PARP to its cleaved form in a time-dependent manner (Figure 10A, 10B and 10C). The balance between the expression levels of the Bcl-2 family proteins, Bcl-2 (anti-apoptotic) and Bax (pro-apoptotic), is critical for cell survival and death as the increase in Bax/Bcl-2 ratio contributes to the release of cytochrome C from mitochondria and activation of intrinsic apoptotic pathway [52]. Figure 10D shows that Bax expression was increased and the Bcl-2 expression was decreased time-dependently. A densitometric analysis of the bands revealed that PRME increased the Bax/Bcl-2 ratio in a time-dependent manner which is responsible for the PRME induced apoptosis in MCF-7 cells. Furthermore, procaspase-8 level is decreased, caspase-8 level is elevated and there was appearance of the t-Bid after the treatment of PRME (Figure 10E and 10F). Previously it is reported that, caspase-8 links intrinsic pathway with extrinsic pathway by cleaving Bid into truncated-Bid and plays important role in activation of both these pathways [53]. These results suggest that PRME induced apoptosis through the regulation of Bax/Bcl-2 ratio and the activation of caspases.

**Figure 10:** Western blot analysis of apoptosis related proteins of MCF-7 cells treated with 300 µg/ml PRME. Graphs adjoining the blots represent the expression levels of corresponding proteins for indicated time intervals: (A) Pro and cleaved caspase-9, (B) Pro and cleaved caspase-3, (C) Native and cleaved PARP, (D) Bax and Bcl-2, (E) Pro and cleaved caspase-8, (F) Bid and t-Bid.

### Identification of Probable Active Compounds and Standardisation of PRME

It is well established that the medicinal properties of lichens are largely attributed to the active compounds present in them and these active compounds are unique to their symbiosis. So, the lichens become the topic of major interest to investigate and explore for their diverse pharmacological applications. Phytochemical analysis of 70% methanolic extract of *P. reticulatum* (PRME) was carried out using standard qualitative and quantitative methods. This study revealed the presence of phenolics, flavonoids and alkaloid in abundant amount however minute quantities of carbohydrates, tannins and ascorbic acid (Table 2) were also present. HPLC analysis was then performed to identify the presence of bioactive compounds by comparing the retention time of reference compounds under the same condition. Four main peaks having retention times 2.4, 3.13, 3.64, 4.68 minutes appeared on the chromatogram of HPLC analysis that were corresponded to the chromatographic patterns of purpurin, catechin, tannic acid and reserpine respectively (Figure 11). These identified compounds were then individually tested for their cytotoxicity against A549, MCF-7 and WI-38 cells. It was found that tannic acid, catechin and purpurin showed effective cytotoxicity against MCF-7 cells while remain negligibly cytotoxic to A549 and WI-38 cells at any of the examined concentration, as corroborated by their IC_50_ values (Table 3) (Figure 12). Reserpine, on the other hand, showed excellent cytotoxicity with a striking IC_50_ against all of the examined cell lines. Since PRME did not show significant cytotoxicity against A549 and WI-38 cells, it may be possible that the low concentration of reserpine (as reflected from HPLC chromatogram) or the presence of other numerous phytochemicals in PRME lessens the cytotoxicity showed by reserpine alone. It was demonstrated that phenolics and flavonoids show their antioxidant feat through scavenging or metal chelating processes [54], [55]. Tannins act as radical scavengers, intercepting active free radicals and also plays a role in treating various degenerative diseases such cancer, multiple sclerosis, atherosclerosis and aging process [56]. Catechin and purpurin are already reported for their effective antioxidant potentials [57], [58]. The anticancer activity of catechin is also well established [59]. On the other hand antioxidant potentials of reserpine and its derivatives are also demonstrated [60]. Reserpine is also found to possess antileukemic action in hybrid male mice [61]. Since the extract is presumably a mixture of several compounds, it may be possible that some compounds are responsible for antioxidant activity and others are responsible for the anticancer activity against MCF-7 cells or these activities were resulted from the synergistic effects of the numerous phytoconstituents present in PRME.

**Figure 11:** HPLC chromatogram of PRME. Inset shows expanded region of the chromatogram with retention time of 4.5–10 minutes. Peaks marked signify the retention peak of purpurin (2.4 min), catechin (3.13 min), tannic acid (3.64 min) and reserpine (4.68 min).

**Figure 12:** Effect of various compounds on cell proliferation and viability of A549, MCF-7 and WI-38 cells. Cells were treated with increasing concentrations of compounds for 48 hours; cell proliferation and viability was determined with WST-1 cell proliferation reagent. Results were expressed as cell viability (% of control). (A) Tannic acid, (B) Catechin, (C) Purpurin, (D) Reserpine. All data is expressed as mean ± SD (n = 6). *p<0.05, **p<0.01 and ***p<0.001 vs. 0 µg/ml.

**Table 2:** Qualitative and quantitative phytochemical analysis of PRME.

	Phytochemicals										
Tests	Phen	Flav	Carbo	Tan	Alka	Asc	Ter	Triter	Anth	Sap	Gly
**Qualitative**	+	+	+	+	+	+	+	+	+	+	+
**Quantitative**	52.47±0.73	30.44±0.15	1.085±0.022	0.233±0.021	67.0±0.66	0.354±0.032	ND	ND	ND	ND	ND

“+” represents presence of the phytoconstituent; “−” represents absence of the phytoconstituent; “ND” represents “Not determined”. Phen- Phenol, Flav- Flavonoid, Carbo- Carbohydrate, Tan.- Tannin, Alka- Alkaloid, Asc- Ascorbic acid, Ter- Terpenoids, Triter- Triterpenoids, Anth-Anthraquinones, Sap- Saponin, Gly- Glycoside; Total phenolics (mg/100 mg extract gallic acid equivalent), Total flavonoids (mg/100 mg extract quercetin equivalent), Carbohydtrate (mg/100 mg extract glucose equivalent), Tannin (mg/100 mg extract catechin equivalent). Alkaloid (mg/100 mg extract reserpine equivalent), Ascorbic acid (mg/100 mg extract L-ascorbic acid equivalent)

**Table 3:** IC_50_ values of tannic acid, catechin, purpurin and reserpine against A549, MCF-7 and WI-38 cells.

Phytochemicals	A549	MCF-7	WI-38
**Tannic acid**	>600	103.31±6.88	>600
**Catechin**	>600	255.79±18.59	>600
**Purpurin**	>600	560.11±78.83	>600
**Reserpine**	65.29±2.27	46.78±1.31	44.34±1.54

_50_ values are determined in µg/ml. Data expressed as mean ± S.D (n = 6).^#^ All the IC

## Conclusions

The findings of this study support that the 70% methanolic extract of *P. reticulatum* is considerably an effective radical scavenger indicating the presence of many natural antioxidants or active compounds. Flow cytometric and western blotting studies proposed that PRME induced cell cycle arrest and apoptosis in MCF-7 cells. These outcomes suggest that the different pathways are involved in the anticancer activity of *P. reticulatum* against MCF-7 cells (Figure 13), and there is a need to characterize the bioactive compounds responsible for these activities. Furthermore, extensive *in vivo* research with xenograft and pre-clinical models with those compounds will justify its use in combination therapy and novel drug delivery systems, thus making it a promising candidate for management of breast cancer patients.

**Figure 13:** Proposed mechanisms of PRME-induced S and G2/M phase cell cycle arrest and apoptosis in MCF-7 cells.
